The article "Antidiabetic, antioxidant, antihyperlipidemic effect of extract of Euryale ferox salisb. with enhanced histopathology of pancreas, liver and kidney in streptozotocin induced diabetic rats" was retracted in 2023. Reasons: manipulated images; duplicated images; lack of ethics approval or compliance; concerns about the images.

# Antidiabetic, antioxidant, antihyperlipidemic effect of extract of *Euryale ferox salisb*. with enhanced histopathology of pancreas, liver and kidney in streptozotocin induced diabetic rats

**DOI:** 10.1186/s40064-015-1059-7

**Published:** 2015-07-03

**Authors:** Danish Ahmed, Vikas Kumar, Amita Verma, Girija Shankar Shukla, Manju Sharma

**Affiliations:** Department of Pharmaceutical Sciences, Faculty of Health Sciences, Sam Higginbottom Institute of Agriculture, Technology and Sciences (SHIATS)-Deemed University, Allahabad, India; Department of Pharmacology, Faculty of Pharmacy, Jamia Hamdard, New Delhi, India; Faculty of Health Sciences, Sam Higginbottom Institute of Agriculture, Technology and Sciences (SHIATS)-Deemed University, Allahabad, India; Department of Pharmacology, Hamdard Institute of Medical Sciences and Research (HIMSR), Jamia Hamdard, New Delhi, India

**Keywords:** *Euryale ferox salisb*. diabetes, Hyperlipidemia, Oxidative stress

## Abstract

**Background:**

Ethanolic extract of *Euryale ferox salisb*. (EFx) may have an effect on the activity of hepatic antioxidant enzymes, glycemic control and lipid profile and histopathology of pancreas, liver and kidney of streptozotocin (STZ)—induced diabetic wistar rats.

**Methods:**

Wistar albino rats were divided into eight groups viz. non-diabetic (normal control), diabetic control (STZ-induced), diabetic treated (infused with different doses of *Euryale ferox. Salisb.* ethanolic extract) and diabetic conventional treated (treated with Glibenclamide). Diabetes was induced by administering streptozotocin (60 mg/kg body weight) intraperitoneal (i.p). The ethanolic extract was supplemented in different doses through oral route. Biochemical investigations were carried out according to previously reported methods. Histopathological examinations were done accordingly.

**Results:**

The EFx supplemented diabetic rats significantly (p < 0.001) decreased the blood glucose level in a dose dependent manner. Plasma insulin level was significantly increased in EFx treated rats. The hepatic gluconeogenic enzymes activities were restored to normal in EFx treated rats. Activities of superoxide dismutase (SOD), catalase (CAT), glutathione peroxidase (GPx) and reduced glutathione (GSH) were significantly increased (p < 0.001) among EFx treated rats. Lipid profile was reinstated to nearly normal level among EFx treated rats. Histopathological investigations revealed that microscopic architecture of pancreatic, hepatic and renal cells improvised in EFx treated diabetic rats.

**Conclusion:**

EFx supplement could improve the glycemic control as well as lipid profile in diabetic rats along with improvised antioxidant enzymes which has beneficial effect in preventing the diabetic complications by scavenging the free radicals in diabetic rats.

## Background

There are several evidences that demonstrate that diabetic complications are closely associated with oxidative stress persuaded by free radicals generation (Pitkänen et al. 1992) Type-2 diabetes mellitus (T2DM) is a multi-functional disease which is associated with hyperglycemia and lipoprotein abnormalities (Ugochukwu and Babady 2002). Damage to the cell, in turn results in the enhancement of reactive oxygen species (ROS) production. Abnormally high level of ROS has been found to play an important role in causation of the development and pathogenesis of T2DM. Free radicals easily formed during diabetic state, serves an important role in the genesis of diabetic complications (Ahmed et al. 2014a).

Antioxidant enzymes such as superoxide dismutase (SOD), catalase (CAT), glutathione peroxidase (GPx) and reduced glutathione (GSH) provides an important assistance in scavenging the free radicals by breaking down the ROS. Prior researches have reported that a defect in the ROS scavenging machinery in T2DM patients as compared to the normal control (Ahmed et al. 2013).

Disturbances in the lipid profile is so high that diabetes has been called “more a disease of lipid than carbohydrate metabolism” (Rawi et al. 1998). Levels of total cholesterol (TC), triglycerides (TG), low density lipoprotein cholesterol (LDL-c) were increased to a momentous level in T2DM. In contrast the level of high density lipoprotein cholesterol (HDL-c) was significantly reduced in T2DM (Ahmed et al. 2014b; Kumar et al. 2013a, b).

Due to the competence of antioxidants to assuage oxidative stress in cells and its contribution in helping to prevent diabetic complications, the chase for antioxidants in the past decades has attracted much interest and many plants have been discovered to have great antioxidant potential. *Euryale ferox salisb*. is an aquatic plant that belongs to family nymphaeaceae. It is also known as fox nut or gorgon nut. It is mainly distributed in East Asia to China to North and North East India. *Eurylae ferox salisb*. produces starchy white seeds which are edible. In India, the processed white seeds of *Euryale ferox salisb*. is known as Makhana. Leaves of E.Ferox salisb. are used in condition of difficult parturition (Duke and Ayensu 1985). Further, E.Ferox salisb. has also been used as traditional oriental medicine to treat various ailments including kidney failure, diarrhea and spleen dysfunction. Recent research studies indicate that *E. Ferox salisb*, seeds could reduce the myocardial ischemic reperfusion injury (Das et al. 2006). One of the recent study explores the antioxidant activities of the isolated compounds from *E. Ferox Salisb*. seeds (Song et al. 2011). The mechanism of action of STZ to induce diabetes is its selective toxicity to pancreatic β-cells via generation of NO free radicals. (Moncada et al. 1991). It is well known that the activity of free radical scavenging compounds i.e. antioxidant enzymes is very low in the islet of langerhans of pancreas as compared to the other tissues (Gandy et al. 1981). On the basis of antioxidant activity of the *E. Ferox salisb*. seeds, we aimed to investigate the plausible role of EFx on STZ-induced diabetic rats.

Thus, the present study was carried out to investigate the effect of ethanolic extract of *E. Ferox salisb.* on the carbohydrate metabolism, glycemic control, insulin level, hepatic gluconeogenic enzymes, renal function parameters and antioxidant enzymes level in conjunction with the pathological corrections in architecture of pancreas, liver and kidney.

## Methods

### Experimental animals

Healthy adult male albino Wistar rats, bred and reared at Indian Institute of Toxicological Research (IITR), Lucknow were used for purpose of the experimentation. Weight-matched animals (140–160 g) were selected and housed in polypropylene cages layered with husk and kept in a semi-natural light/dark condition (12 h light/12 h dark). The animals were allowed free access to water and standard pellet diet (Amrut Feeds, Pune, India). 

### Chemicals, reagents and biochemical estimation kits

Hexokinase, glucose-6-phosphate dehydrogenase, glucose-6-phosphatase, fructose-1-6-bisphosphate were purchased from Sigma Aldrich (India). Blood glucose, lipid profile, and antioxidant enzymes kits were purchased from Span Diagnostics, Surat (India). Streptozotocin was purchased from Sigma Aldrich (India). Other needed chemicals used in the study were procured either from Sigma Aldrich (India) or CDH Mumbai (India).

### Induction of diabetes

Wistar rats were injected intraperitoneally with STZ dissolved in 0.1 M citrate buffer (pH = 6.5) at 60 mg/kg. Animals of control group received equal volume of vehicle. After 48 h of STZ injection, blood glucose level of the diabetes induced rats was estimated. The rats depicting values ranging FBG ≥ 230 mg/dL, were considered to be diabetic.

### Preparation of extracts

Extract of *Euryale ferox salisb*. seeds was prepared according to guideline of Lee et al. (Lee et al. 2002). Dried powder (100 g) of *E. Ferox salisb.* seeds was placed in a conical flask with 70% ethanol and extracted at 80°C for 3 h. The filtration of the extract was performed along with the concentration of the extract by rotary evaporator (Buchi, India) under low pressure. The resultant residue was freeze dried and stored at −70°C. After freeze drying the whole extract was eluted with *n*-hexane, dichloromethane, ethyl acetate and n-butanol in a stepwise manner. After the sequential screening of the extract, the resultant fractions were collected and the remaining solvents were removed by rotary evaporation. The powder (dried) was dissolved in dimethyl sulfoxide (DMSO) and diluted with phosphate buffered saline (pH = 7.4). The percentage yield of the crude extract was calculated to be 3.17%.

### Administration of plant extracts

The extract of the parts of *Euryale Ferox Salisb*. (EFx) was administered to the rats through force-feeding gastric gavage route. This was executed by inserting an infant oral feeding tube, which was connected to a syringe containing the extract, into the gastric region of the rat. The animals were fasted 30 min before and after the treatment to ensure maximum bioavailability (Sridhar et al. 2005).

### Preliminary study—determining the dosage for crude drug

One week after the induction of diabetes, rats with blood glucose level >250 mg/dL, were subjected to fasting for 16 h. They were divided into different groups, with five rats in each group. *N*-hexane, di-chloromethane, ethyl acetate, *n*-butanol and aqueous extract ranging from 100 to 800 mg/kg body weight, were administered to the animals and blood glucose was determined at the end of 5 h after the oral administration of the extracts (Karunanayake et al. 1984). The lowest dose that brought about the maximum antihyperglycemic effect for each plant extract was given through oral intubations for the repeated administration. The effective dose of all the extracts was found to be 400 mg/kg body weight. The selected doses of the plant extracts were given on everyday till completion of the experiment (i.e., 45 days).

### Repeated administration of *E. Ferox salisb*. seeds extract (EFx)

After a week of induction of diabetes in albino rats, fasting blood glucose levels of fasted rats was measured (Ahmed et al. 2014a). Rats with plasma glucose level more than >250 mg/dL were included in the study. Rats were divided into seven groups of five each. Groups 1 and 2, viz, normal and diabetic control rats received vehicle alone [0.1% dimethyl sulfoxide (DMSO) 1 ml/kg body weight]. Groups 3–6 were treated with the effective dose of *n*-hexane, di-chloromethane, ethyl acetate, *n*-butanol and water extracts dissolved in vehicle solution through oral route for 15 days, respectively. Group 7 was treated with insulin (3-IU/kg) for 15 days. Blood samples were collected periodically. At the end of the repeated administration of the drug, the collected blood samples were analyzed for any toxic effect. Different doses of extract did not show any significant difference in the food consumption and body weight when compared to the normal rats. There was no lethality and toxicity found with any dose till the completion of the experiment. Therefore, the conclusion was that 400 mg/kg body weight was safe to use.

### Experimental design

A total of 35 male albino wistar rats were utilized and were randomly divided into 7 groups of 5 animals in each group:

- Group I—Normal rats (untreated with dimethylsulfoxide, [DMSO].
- Group-II—Diabetic control (administered with Streptozotocin (STZ).
- Group-III—Diabetic control + EFx seed extract (EFx) (100 mg/kg body weight).
- Group-IV—Diabetic control + EFx seed extract (EFx) (200 mg/kg body weight).
- Group-V—Diabetic control + EFx seed extract (EFx) (300 mg/kg body weight).
- Group-VI—Diabetic control + EFx seed extract (EFx) (400 mg/kg body weight).
- Group-VII—Diabetic control + Glibenclamide (1 mg/kg body weight).

The extract was administered to the respective groups through oral route using intragastric tube for 45 days.

### Biochemical evaluation

Rats of the different groups were kept on fasting overnight and the blood was withdrawn by retro orbital puncture under light anesthesia. Blood was withdrawn from the rats on the 1st, 22nd and 45th day after the induction of diabetes to assess the blood glucose and plasma insulin level by glucose oxidase method (Kesari et al. 2005) and modified method of Herbert (Herbert et al. 1965) respectively. The alteration in the body weight was observed throughout the therapy in the experimental animals.

Oral glucose tolerance test (OGTT) was performed according to the method described by Kumar et al. (2013). OGTT was evaluated to determine the effect of EFx on peripheral utilization of glucose in normal rats. Wistar-albino rats were grouped into 7 groups (n = 5). All the rats were administered with different doses of EFx and Glibenclamide for 30 min. On completion of 30 min all the groups received 2 g/kg of glucose by oral route. The blood samples were collected at regular time period of 0, 0.5, 1.0, 1.5 and 2.0 h to estimate the oral glucose tolerance. At the termination of treatment i.e. after 45 days, animals were deprived of food for overnight. Activities of hepatic hexokinase, glucose-6-phsophatase, fructose-1-6-bisphosphatase, glucose-6-phosphate dehydrogenase were assayed according to the method of Branstrup (1957), method of Koide and Oda (1959), method of Gancedo (1971) and method of Robert (1966), respectively.

The level of the hexokinase was determined by the using reported method with minor modification (Branstrup et al. 1957). The liver tissue was thawed, weighed and homogenized in ice-cold 0.1 M phosphate-buffered saline (pH 7.4) to a concentration of 50 mg/ml. The assay mixture contains the 7.5 mM MgCl2, 3.7 mM glucose, 11 mM thioglycerol and 45 mM HEPES (4-(2-hydroxyethyl)-1-piperazineethanesulfonic acid) buffer. Assay mixture 0.9 ml added into the culvert and 0.3 ml of 0.22 M ATP added and mixed well. After that, 0.1 ml of the tissue supernatant was added into the culvert and determinations of the absorbance at 340 nm the hexokinase activity as units/min/mg of protein of tissue was recorded. The level of the glucose-6-phosphatase activity was measured according reported method of Koide et al. with minor modification (Koide and Oda 1959). Liver tissue was homogenate in ice-cold 0.1 M phosphate buffer saline (pH 7.4) to a concentration of 50 mg/ml. 0.1 ml of 0.1 M glucose-6-phosphatase solution and 0.3 ml of 0.5 M maleic acid buffer (pH 6.5) was mixed in a test tube and incubated at 370°C for 15 min. The reaction was stopped by adding 1 ml of 10% trichloroacetic acid, followed by chilling in ice, after stopping reaction the mixture was centrifuged at 3000 rpm for 10 min. The absorbance was measured at the 340 nm and expressed of the glucose-6-phosphatase at the liberation of the inorganic phosphate units/min/mg of protein of tissue. The level of the fructose-1,6-bisphosphatase was estimated by using the reported method with minor modification (Gancedo and Gancedo 1971). Liver tissue was homogenized in ice-cold 0.1 M phosphate buffer saline (pH 7.4). The assay mixture containing the 1.2 ml of trise HCl buffer (0.1 M, pH 7.0), 0.1 ml of substrate (0.05 M), 0.25 ml of MgCl2 (0.1 M), 0.1 ml of KCl (0.1 M), 0.25 ml of ethylenediaminetetraacetic acid (0.001 M) solution and 0.1 ml of enzyme homogenate and maintained the final sample volume 2 ml. The mixture was incubated for 15 min at 370°C. The 10% solution of the trichloroethanoic acid was used for the termination of the reaction. The reaction mixture was centrifuged and the supernatant was used for the phosphorous estimation). In the supernatant, the 1 ml of ammonium molybdate and 0.4 ml of amino naphthol sulfonic acid were added. The blue color developed after 20 min and measurement of the absorbance at 680 nm was done. The activity of the fructose-1,6-bisphosphatase measured in units/min/mg of protein.

The lipid parameters viz. total cholesterol, HDL cholesterol and triglycerides were evaluated according the methods of Zlatkis (1953), Burnstein (1970) and Foster and Dunn (1973), respectively. Level of serum LDL cholesterol and VLDL cholesterol were estimated according to the Friedewald formula (Friedewald et al. 1972). Hepatic glycogen level was assessed by the method given by Kemp (1954). The levels of lipid peroxidation (LPO) in the tissues were evaluated by the method of Ohkawa (1979). Level of superoxide dismutase (SOD) was assayed by the method of Kakkar (1984). The level of catalase (CAT) enzyme was evaluated by the method given by Sinha (1972). Glutathione Peroxidase (GSH-Px) was assayed by the method given by Rotruck (1973). Level of reduced glutathione (GSH) was assessed by the method of Ellman (1959).

### Production of liver and kidney homogenate

For the estimation of the antioxidant level, the rats of the respective groups were kept on fasting overnight. All the rats were decapitated and an abdominal incision was performed, in order to harvest liver and pancreas. The whole organs were thoroughly cleaned with chilled normal saline on ice. A 10% (w/v) homogenate of the liver and pancreas (0.03 M sodium phosphate buffer, pH-7.4) was prepared with the help of Ultra-Turrax homogenizer maintaining the speed at 9500 rpm.

### Observation of general condition of rats

The overall general condition of rats such as psychological activity, food intake, water intake, urine output, general locomotion, and skin was observed every day. The parameters such as body weight and food intake were determined for every week.

### Histological assessment of liver, kidney, pancreas and heart sample by Heamatoxylin Eosin (H/E) staining

At the end of the therapy, all the rats of different groups were sacrificed using mild anesthesia. After collection of the blood samples, the liver, kidney, pancreas and heart tissues were fixed in neutral formalin solution for 48 h, dehydrated by passing through graded series of alcohol embedded in paraffin blocks. 4 µm thick sections were prepared using a semi-automated rotator microtome.

### Statistical analysis

Statistical analysis was performed using GRAPH PAD Prism software package, Version 5.0. All the data were expressed as mean ± standard error mean (SEM). The comparisons within groups was evaluated utilizing independent student *T* test and one way analysis of variance (ANOVA). The value of p < 0.05 or p < 0.01 was considered to be statistically significant.

## Results

### Effect of EFx on blood glucose level in normal and STZ induced diabetes treated rats

The biochemical parameters of glycemic control in the animals has been summarized in Table 1 (Figure 1). The intraperitoneal administration of streptozotocin (STZ) resulted in nearly fourfold increase of the fasting blood glucose levels in the male/female diabetic Wistar rats. The blood glucose level was measured at different time intervals during the research exertion viz. on the very first day of induction of diabetes, at the middle of the study i.e. on 21st day and at the end of the experiment i.e. on 45th day. It was observed that with the gradual increase in dose of the EFx, the blood glucose level was improvised. At the end of 45 days period, EFx treated diabetic animals showed a significant reduction of blood glucose level nearly to the normal level compared with the diabetic animals (p < 0.05).

**Table 1:** Effect of *Euryale ferox salisb.* seeds extract (EFx) on blood glucose level in normal and STZ induced diabetic treated rats

Groups	Blood glucose level in mg/dL at different time intervals during experimentation		
	At start (on 1st day)	On 21st day	On 45th day
Normal rats [untreated with dimethylsulfoxide, (DMSO)] Group 1	82.38 ± 0.6308^a^	82.25 ± 0.2649^a^	81.80 ± 0.4055^a^
Diabetic control [administered with streptozotocin (STZ)] Group 2	303.8 ± 0.9011^b^	310.5 ± 0.2231^b^	312.5 ± 0.4212^b^
Diabetic + (EFx) (100 mg/kg body weight) Group 3	301.0 ± 0.2698	264.1 ± 1.152	201.7 ± 0.3738
Diabetic + (EFx) (200 mg/kg body weight) Group 4	297.8 ± 0.3096	235.4 ± 0.8799	173.1 ± 0.8970
Diabetic + (EFx) (300 mg/kg body weight) Group 5	295.4 ± 0.3857	184.0 ± 0.6072	107.6 ± 1.422^**^
Diabetic + (EFx) (400 mg/kg body weight) Group 6	293.6 ± 0.3771	146.7 ± 0.5004	91.08 ± 0.5402^***^
Diabetic + glibenclamide (1 mg/kg body weight) Group 7	290.9 ± 0.2182	117.4 ± 1.004^**^	83.14 ± 0.6532^***^

The data are expressed as mean ± SEM (n = number of animals in each group = 5). The comparisons has been made by one way ANOVA followed by Dunnent’s test.

*ns* non-significant, *STZ* Streptozotocin.

* p < 0.05 is considered as significant when compared to the control group (0 h).

** p < 0.001 is considered as very significant when compared to the control group (0 h).

*** p < 0.001 is considered as extremely significant when compared to the control group (0 h).

^a^Compared to diabetic control.

^b^Compared to normal control.

**Figure 1:** Effect of EFx on blood glucose level at different time interval of therapy, Group 1: normal control; Group 2: STZ (60 mg/kg i.p.); Group 3: diabetic control + (EFx) (100 mg/kg body weight); Group 4: diabetic control + (EFx) (200 mg/kg body weight) and continue for 45 days; Group5: diabetic + diabetic control + (EFx) (300 mg/kg body weight) and continue for 45 days; Group 6: diabetic control + (EFx) (400 mg/kg body weight) and continue for 45 days; Group 7: diabetic control + glibenclamide (1 mg/kg body weight) and continue for 45 days.

### Effect of EFx on plasma insulin level in normal and STZ induced diabetes treated rats

The level of plasma insulin was measured at different periods during the experimentation. A significant decrease in the level of plasma insulin was observed in the untreated diabetic rats compared to the normal rats and the level of plasma insulin was further decreased in the untreated diabetic rats at the end of the study i.e. after 45 days. Treatment with the methanol/dichloromethane extract of EFx in a dose dependent manner. Treatment with 400 mg/kg body weight of EFx was shown to produce most significant (p < 0.05) effect on the level of plasma insulin. It amplified the level of plasma insulin nearly to the normal as compared to the other doses of EFx at the end of research exertion (Table 2; Figure 2).

**Table 2:** Effect of *Euryale ferox salisb.* seed extract (EFx) on plasma insulin level in normal and STZ induced and treated diabetic rats

Groups	Plasma insulin level in µM at different time interval of experimentation		
	At start (on 1st day)	On 21st day	On 45th day
Normal rats [untreated with dimethylsulfoxide, (DMSO)] Group 1	12.22 ± 0.2028^a^	12.37 ± 0.1772^a^	12.39 ± 0.1154^a^
Diabetic control [administered with Streptozotocin (STZ)] Group 2	3.710 ± 0.1482^b^	3.136 ± 0.01208^b^	3.034 ± 0.02482^b^
Diabetic + (EFx) (100 mg/kg body weight) Group 3	4.260 ± 0.1040	5.812 ± 0.03929	6.822 ± 0.02596
Diabetic + (EFx) (200 mg/kg body weight) Group 4	4.250 ± 0.02168	6.028 ± 0.005831	7.936 ± 0.02542
Diabetic + (EFx) (300 mg/kg body weight) Group 5	4.806 ± 0.03655	7.058 ± 0.03277	9.496 ± 0.1394^**^
Diabetic + (EFx) (400 mg/kg body weight) Group 6	4.896 ± 0.02786	9.136 ± 0.04854^**^	11.66 ± 0.1689^***^
Diabetic + glibenclamide (1 mg/kg body weight) Group 7	5.058 ± 0.03382	9.734 ± 0.09304^**^	12.34 ± 0.1080^***^

The data are expressed as mean ± SEM (n = number of animals in each group = 5). The comparisons has been made by one way ANOVA followed by Dunnent’s test.

*ns* non-significant, *STZ* Streptozotocin.

* p < 0.05 is considered as significant when compared to the control group (0 h).

** p < 0.001 is considered as very significant when compared to the control group (0 h).

*** p < 0.001 is considered as extremely significant when compared to the control group (0 h).

^a^ Compared to diabetic control.

^b^Compared to normal control.

**Figure 2:** Effect of EFx on plasma insulin level at different time interval of therapy, Group 1: normal control; Group 2: STZ (60 mg/kg i.p.); Group 3: diabetic control + (EFx) (100 mg/kg body weight); Group 4: diabetic control + (EFx) (200 mg/kg body weight) and continue for 45 days; Group5: diabetic + diabetic control + (EFx) (300 mg/kg body weight) and continue for 45 days; Group 6: diabetic control + (EFx) (400 mg/kg body weight) and continue for 45 days; Group 7: diabetic control + glibenclamide (1 mg/kg body weight) and continue for 45 days.

### Effect of EFx on OGTT in normal and STZ induced (treated) diabetic rats during 120 min (2 h)

The results from the research exertion clearly indicate that the of methanol/dichloromethane extract of Albizzia Lebbeck Benth. stem bark (EFx) (400 mg/kg body weight) and Glibenclamide (1 mg/kg) reduced the blood glucose level (significant hyperglycemia due to administration of glucose load of 2 g/kg p.o to a significant level (p < 0.05) after 2 h of oral administration as compared to the diabetic control group (Table 3; Figure 3).

**Table 3:** Effect of *Euryale ferox salisb.* seeds extract (EFx) during 120 min (2 h) on OGTT in normal and STZ induced diabetic (treated) rats

Groups	Time (h)				
	0 h	0.5 h	1 h	1.5 h	2 h
Normal rats [untreated with dimethylsulfoxide, (DMSO)] Group 1	82.91 ± 0.3829^a^	95.60 ± 0.2651^a^	108.62 ± 0.3387^a^	117.67 ± 0.9812^a^	138.15 ± 0.4991^a^
Diabetic control (administered with Streptozotocin (STZ) Group 2	265.9 ± 0.9826^b^	278.2 ± 0.8519^b^	284.7 ± 0.2911^b^	279.1 ± 0.8171^b^	274.9 ± 0.3012^b^
Diabetic + (EFx) (100 mg/kg body weight) Group 3	235.0 ± 1.086	225.0 ± 0.8882	221.0 ± 0.2465	203.9 ± 0.8683	182.4 ± 0.2997
Diabetic + (EFx) (200 mg/kg body weight) Group 4	225.2 ± 0.9767	214.8 ± 0.8538	212.4 ± 0.2989	198.0 ± 0.6565	171.6 ± 0.4256
Diabetic + (EFx) (300 mg/kg body weight) Group 5	214.2 ± 1.263	211.5 ± 0.6072	202.8 ± 0.4556	185.7 ± 1.784	142.8 ± 0.7964^**^
Diabetic + (EFx) (400 mg/kg body weight) Group 6	203.1 ± 1.652	192.3 ± 0.5702	182.8 ± 0.3597	162.4 ± 0.4513^*^	88.45 ± 0.7672^***^
Diabetic + glibenclamide (1 mg/kg body weight) Group 7	198.3 ± 0.5980	182.4 ± 0.5737	170.9 ± 0.3304	141.7 ± 0.5050^**^	82.80 ± 0.5378^***^

The data are expressed as mean ± SEM (n = number of animals in each group = 5). The comparisons has been made by one way ANOVA followed by Dunnent’s test.

*ns* non-significant, *STZ* Streptozotocin.

* p < 0.05 is considered as significant when compared to the control group (0 h).

** p < 0.001 is considered as very significant when compared to the control group (0 h).

*** p < 0.001 is considered as extremely significant when compared to the control group (0 h).

^a^Compared to diabetic control.

^b^Compared to normal control.

**Figure 3:** Effect of EFx on oral glucose tolerance test (OGTT) during 120 min (2 h) of therapy, Group 1: normal control; Group 2: STZ (60 mg/kg i.p.); Group 3: diabetic control + (EFx) (100 mg/kg body weight); Group 4: diabetic control + (EFx) (200 mg/kg body weight) and continue for 45 days; Group 5: diabetic + diabetic control + (EFx) (300 mg/kg body weight) and continue for 45 days; Group 6: diabetic control + (EFx) (400 mg/kg body weight) and continue for 45 days; Group 7: diabetic control + glibenclamide (1 mg/kg body weight) and continue for 45 days.

### Effect of EFx weight variation (grams) in normal and STZ induced diabetic (treated) rats

The body weight variation of the rats was observed at the beginning and end of the research exertion. As it is obvious from the table (Table 4; Figure 4), that weight of the diabetic (untreated) rats was reduced to a significant level. Weight of the EFx treated rats was increased to a momentous level (p < 0.05) as compared to the weight of normal rats.

**Table 4:** Effect of *Euryale ferox salisb.* seeds extract (EFx) on body weight variation (grams) in normal and STZ induced diabetic treated rats

Groups	Time (h)	
	1st day	45th day
Normal rats [untreated with dimethylsulfoxide, (DMSO)] Group 1	263.6 ± 0.8124^a^	265.0 ± 1.673^a^
Diabetic control [(administered with Streptozotocin (STZ)] Group 2	213.8 ± 1.594^b^	210.8 ± 0.4899^b^
Diabetic + (EFx) (100 mg/kg body weight) Group 3	217.0 ± 1.140	222.8 ± 1.655
Diabetic + (EFx) (200 mg/kg body weight) Group 4	220.6 ± 0.2449	234.2 ± 1.463
Diabetic + (EFx) (300 mg/kg body weight) Group 5	222.6 ± 0.5099	237.6 ± 0.5099
Diabetic + (EFx) (400 mg/kg body weight) Group 6	226.2 ± 0.8000	252.6 ± 1.631^**^
Diabetic + glibenclamide (1 mg/kg body weight) Group 7	227.0 ± 0.9487	262.0 ± 0.7071^***^

The data are expressed as mean ± SEM (n = number of animals in each group = 5). The comparisons has been made by one way ANOVA followed by Dunnent’s test.

*ns* non-significant, *STZ* Streptozotocin.

* p < 0.05 is considered as significant when compared to the control group (0 h).

** p < 0.001 is considered as very significant when compared to the control group (0 h).

*** p < 0.001 is considered as extremely significant when compared to the control group (0 h).

^a^ Compared to diabetic control.

^b^Compared to normal control.

**Figure 4:** Effect of EFx on body weight variation at different time interval of therapy, Group 1: normal control; Group 2: STZ (60 mg/kg i.p.); Group 3: diabetic control + (EFx) (100 mg/kg body weight); Group 4: diabetic control + (EFx) (200 mg/kg body weight) and continue for 45 days; Group 5: diabetic + diabetic control + (EFx) (300 mg/kg body weight) and continue for 45 days; Group 6: diabetic control + (EFx) (400 mg/kg body weight) and continue for 45 days; Group 7: diabetic control + glibenclamide (1 mg/kg body weight) and continue for 45 days.

### Effect of EFx on hepatic enzymes in normal and STZ induced diabetic treated rats

Table 5 (Figure 5) portrays the alteration in the activities of carbohydrate metabolizing enzymes in the liver of diabetic control group and other groups of experimental animals. The activities of hepatic hexokinase and glucose-6-phosphate dehydrogenase (G6PD) were found to be decreased. On the other hand, the level of gluconeogenic enzymes viz. glucose-6-phosphatase and fructose-6-phosphatase were significantly increased in the diabetic animals compared to those in normal rats. Administration of different doses of EFx among diabetic rats reversed the alterations in the hepatic enzymes such that animals received 400 mg/kg body weight showed the significant improvement (p < 0.05) in all the hepatic enzymes alterations as compared to the other doses.

**Table 5:** Effect of Euryale *ferox salisb.* seeds extract (EFx) on hepatic enzymes in normal and STZ induced diabetic treated rats

Groups	Biochemical parameters of hepatic enzymes			
	Hepatic hexokinase (units/min/mg of protein)	Gluocse-6-phosphatase (units/min/mg of protein)	Fructose 1-6-biphosphatase (units/min/mg of protein)	Glucose-6-phosphate dehydrogenase (units/min/mg of protein)
Normal rats [untreated with dimethylsulfoxide, (DMSO)] Group 1	0.2360 ± 0.007483^a^	0.0356 ± 0.0002449^a^	0.0320 ± 0.0004472^a^	0.1620 ± 0.003742^a^
Diabetic control (administered with Streptozotocin (STZ) Group 2	0.0880 ± 0.003742^b^	0.0646 ± 0.002249^b^	0.0664 ± 0.0009274^b^	0.0714 ± 0.0006782^b^
Diabetic + (EFx) (100 mg/kg body weight) Group 3	0.1080 ± 0.003742	0.0602 ± 0.0004899	0.0584 ± 0.0007483	0.0754 ± 0.0012080
Diabetic + (EFx) (200 mg/kg body weight) Group 4	0.1400 ± 0.003162	0.0548 ± 0.0005831	0.0526 ± 0.0014	0.0822 ± 0.00080000
Diabetic + (EFx) (300 mg/kg body weight) Group 5	0.1800 ± 0.003162	0.0464 ± 0.0009274	0.0466 ± 0.001030	0.08808 ± 0.01949
Diabetic + (EFx) (400 mg/kg body weight) Group 6	0.2024 ± 0.0006782^**^	0.0408 ± 0.0003742^**^	0.0376 ± 0.0005099^***^	0.1340 ± 0.0050990^**^
Diabetic + glibenclamide (1 mg/kg body weight) Group 7	0.2220 ± 0.003742^***^	0.0532 ± 0.001497^**^	0.0454 ± 0.002315^**^	0.1144 ± 0.003919^**^

The data are expressed as mean ± SEM. (n = number of animals in each group = 5). The comparisons has been made by one way ANOVA followed by Dunnent’s test

*ns* non-significant, *STZ* Streptozotocin.

* p < 0.05 is considered as significant when compared to the control group (0 h).

** p < 0.001 is considered as very significant when compared to the control group (0 h).

*** p < 0.001 is considered as extremely significant when compared to the control group (0 h).

^a^Compared to diabetic control.

^b^Compared to normal control.

**Figure 5:** Effect of EFx on various hepatic enzymes at the end of therapy, Group 1: normal control; Group 2: STZ (60 mg/kg i.p.); Group 3: diabetic control + (EFx) (100 mg/kg body weight); Group 4: diabetic control + (EFx) (200 mg/kg body weight) and continue for 45 days; Group 5: diabetic + diabetic control + (EFx) (300 mg/kg body weight) and continue for 45 days; Group 6: diabetic control + (EFx) (400 mg/kg body weight) and continue for 45 days; Group 7: diabetic control + glibenclamide (1 mg/kg body weight) and continue for 45 days.

### Effect of EFx on serum lipid profile in normal and STZ induced among diabetic (treated) rats

As Evident from the Table 6 that diabetic rats exhibited significant increase in serum total cholesterol, VLDL cholesterol, LDL cholesterol, triglycerides levels and decreased level of HDL cholesterol and hepatic glycogen. Lipid profile of the EFx treated diabetic rats was significantly improved (p < 0.05) as compared to the untreated diabetic rats (Figure 6).

**Table 6:** Effect of *Euryale ferox salisb.* seeds extract (EFx) on lipid profile in normal and STZ induced and diabetic (treated) rats

Groups	Serum lipid profile				
	Total cholesterol (TC) (mg/dL)	HDL cholesterol (HDL-c) (mg/dL)	LDL cholesterol (LDL-c)	Triglycerides (TG) (mg/dL)	Hepatic glycogen (mg glucose equivalents/mg wet tissue)
Normal rats [untreated with dimethylsulfoxide, (DMSO)] Group 1	137.7 ± 1.315^a^	63.19 ± 0.4878^a^	23.54 ± 0.5120^a^	67.57 ± 0.5943^a^	55.70 ± 1.523^a^
Diabetic control [(administered with Streptozotocin (STZ)] Group 2	283.0 ± 0.7544^b^	16.65 ± 0.1162^b^	114.6 ± 0.5353^b^	203.7 ± 0.8567^b^	15.61 ± 0.1631^b^
Diabetic + (EFx) (100 mg/kg body weight) Group 3	231.8 ± 0.3189	24.83 ± 0.4556	92.14 ± 0.2920	184.7 ± 0.6979	20.97 ± 0.2149
Diabetic + (EFx) (200 mg/kg body weight) Group 4	198.1 ± 0.4720	36.27 ± 0.5386	71.43 ± 0.4485	141.6 ± 0.5797	34.01 ± 0.7427
Diabetic + (EFx) (300 mg/kg body weight) Group 5	172.8 ± 0.3100	42.49 ± 0.7798	53.04 ± 0.2755	111.3 ± 0.4677	42.61 ± 0.4618
Diabetic + (EFx) (400 mg/kg body weight) Group 6	151.4 ± 0.4808^***^	58.34 ± 0.5236^***^	32.03 ± 0.5791^**^	74.77 ± 1.225^**^	51.68 ± 0.3041^***^
Diabetic + glibenclamide (1 mg/kg body weight) Group 7	165.7 ± 0.5246^**^	41.62 ± 0.2302^**^	47.58 ± 0.4332^**^	91.99 ± 0.5388^**^	55.79 ± 0.9709^**^

The data are expressed as mean ± SEM (n = number of animals in each group = 5). The comparisons has been made by one way ANOVA followed by Dunnent’s test.

*ns* non-significant, *STZ* Streptozotocin.

* p < 0.05 is considered as significant when compared to the control group (0 h).

** p < 0.001 is considered as very significant when compared to the control group (0 h).

*** p < 0.001 is considered as extremely significant when compared to the control group (0 h).

^a^ Compared to diabetic control.

^b^Compared to normal control.

**Figure 6:** Effect of EFx on lipid profiles at the end of therapy, Group 1: normal control; Group 2: STZ (60 mg/kg i.p.); Group 3: diabetic control + (EFx) (100 mg/kg body weight); Group 4: diabetic control + (EFx) (200 mg/kg body weight) and continue for 45 days; Group 5: diabetic + diabetic control + (EFx) (300 mg/kg body weight) and continue for 45 days; Group 6: diabetic control + (EFx) (400 mg/kg body weight) and continue for 45 days; Group 7: diabetic control + glibenclamide (1 mg/kg body weight) and continue for 45 days.

### Effect of EFx on oxidative stress parameters in normal and STZ induced diabetic (treated) rats

Table 7 clearly illustrates the effect of EFx on the antioxidant enzymes. A marked reduction was noted in the level of superoxide dismutase (SOD), catalase (CAT), Glutathione Peroxidase (GSH-Px), and reduced glutathione (GSH) in the STZ induced diabetic rats. Administration of EFx at different doses for the 45 days to STZ induced diabetic rats significantly (p < 0.05) increased SOD, CAT, GSH-Px levels with maximum effect seen at 400 mg/kg body weight. The enhanced level of TBARS was reversed to near normal after administration of EFx after administering 400 mg/kg body weight of EFx. It is pertinent to note that the EFx was found to be equipped with the antioxidant effect in a dose dependent manner (Figure 7).

**Table 7:** Effect of *Euryale ferox salisb.* seeds extract (EFx) on oxidative stress parameters in liver of normal and STZ induced diabetic treated rats

Groups	Oxidative stress			
	SOD (units/mg protein)	CAT (µ mol/min/mg protein)	GSH-px ((µ mol/min/mg protein)	GSH (mM/100 g tissue)
Normal rats [untreated with dimethylsulfoxide, (DMSO)] Group 1	12.30 ± 0.1642^a^	82.84 ± 0.6566^a^	13.71 ± 0.1077^a^	53.63 ± 0.1813^a^
Diabetic control [administered with Streptozotocin (STZ)] Group 2	3.670 ± 0.07218^b^	22.28 ± 0.2578^b^	5.274 ± 0.1402^b^	21.98 ± 0.2745^b^
Diabetic + (EFx) (100 mg/kg body weight) group 3	5.726 ± 0.1197	36.09 ± 0.2578	7.628 ± 0.08243	35.30 ± 0.3952
Diabetic + (EFx) (200 mg/kg body weight) Group 4	8.366 ± 0.01965	48.08 ± 0.4018	8.820 ± 0.01304	39.09 ± 0.2614
Diabetic + (EFx) (300 mg/kg body weight) Group 5	9.440 ± 0.1626	68.61 ± 0.2086	10.29 ± 0.2236	43.76 ± 0.4200
Diabetic + (EFx) (400 mg/kg body weight) Group 6	11.47 ± 0.1209^***^	76.68 ± 0.8596^**^	12.64 ± 0.04104^***^	50.91 ± 0.3273^***^
Diabetic + Glibenclamide (1 mg/kg body weight) Group 7	9.608 ± 0.1329^**^	71.70 ± 0.3430^**^	10.53 ± 0.1955^**^	34.52 ± 0.3057^**^

The data are expressed as mean ± SEM (n = number of animals in each group = 5). The comparisons has been made by one way ANOVA followed by Dunnent’s test.

*ns* non-significant, *STZ* Streptozotocin.

* p < 0.05 is considered as significant when compared to the control group (0 h).

** p < 0.001 is considered as very significant when compared to the control group (0 h).

*** p < 0.001 is considered as extremely significant when compared to the control group (0 h).

^a^Compared to diabetic control.

^b^Compared to normal control.

**Figure 7:** Effect of EFx on various antioxidant marker enzymes at the end of therapy, Group 1: normal control; Group 2: STZ (60 mg/kg i.p.); Group 3: diabetic control + (EFx) (100 mg/kg body weight); Group 4: diabetic control + (EFx) (200 mg/kg body weight) and continue for 45 days; Group5: diabetic + diabetic control + (EFx) (300 mg/kg body weight) and continue for 45 days; Group 6: diabetic control + (EFx) (400 mg/kg body weight) and continue for 45 days; Group 7: diabetic control + glibenclamide (1 mg/kg body weight) and continue for 45 days.

### Effect of EFx on histopathology of pancreas, kidney, liver and heart

#### Pancreas

Normal control rats exhibited normal histological architecture. Many rounded normal proportions of islet of langerhans were found all around the pancreatic acini. Prominent nuclei with well arranged lobules with surrounding islet cells, were found among normal control rats (Figure 8). Groups received STZ, demonstrated cellular damage to the pancreatic acini and islets, which showed pancreatic β-cell damage and degeneration with asymmetrical vacuoles. EFx treated STZ induced-DM rats showed marked improvement of the cellular injure as (Figure 9), as evident from the partial restoration of islet cells, reduced β-cell damage, more symmetrical vacuoles and an increase in number of islet cells.

**Figure 8:** Effect of *Euryale ferox salisb* seeds extract (EFx) on histological profile of liver in normal, STZ-induced diabetic untreated and STZ-induced diabetic treated wistar rats (original magnification ×40, DXIT 1200, Nikon, Japan). (1) NLIV: heamatoxylin and eosin (H/E) stained sections of liver of normal control rats showing normal portal triad along with normal hepatocytes with central vein (*yellow arrows*). (2) LSTZ: liver section of rats received streptozotocin depicting destructed portal trial, disarranged hepatocytes and central vein (*red arrows*). (3) LEFx100: section of liver supplemented with 100 mg/kg body weight of EFx portraying improvement in structure of portal triad (*green arrows*). (4) LEFx200: liver section of rats received 200 mg/kg body weight of EFx showing arranged hepatocytes (*green arrows*). (5) LEFx300: section of liver or diabetic rats treated with 300 mg/kg body weight. of EFx depicting arranged central vein (*yellow arrows*). (6) LEFx400: liver of diabetic rat showing normal portal traid, central vein and hepatocytes (*green arrows*). (7) LGLIM: liver section of rat administered with Glibenclamide showing normal microvasculature along with normal hepatocytes (*dark yellow arrows*).

#### Kidney

Morphological features of kidney remained normal in the control group like prominent glomeruli, collecting ducts, tubules and ascending and descending loops. STZ-induced DM group showed presence of crystal deposition on the glomeruli along with destructed glomeruli and infiltration of red blood cells (Figure 8). Groups received the EFx demonstrated reversal of these pathological destructions as apparent by the cells regeneration and removal of crystals deposition.

**Figure 9:** Effect of *Euryale ferox salisb* seeds extract (EFx) on histological profile of pancreas in normal, STZ-induced diabetic untreated and STZ-induced diabetic treated wistar rats (original magnification ×10, DXIT 1200, Nikon, Japan). (1) NPAN: heamatoxylin and eosin (H/E) stained sections of pancreas of normal control rat portraying normal islet of langerhans shown by *yellow arrows*. (2) PSTZ: pancreatic section of streptozotocin induced diabetic rat showing no/destroyed islet of langerhans and beta cells depicted by *red arrows*. (3) PEFx-100: pancreatic section of STZ-induced diabetic rats treated with EFx at 100 mg/kg body weight showing small number of islet of langerhans (*green arrows*). (4) PEFx-200: section of pancreas of STZ-induced diabetic rats treated with EFx at 200 mg/kg body weight portraying increased number of islet of langerhans with small proportions of beta cells (*green arrows*). (5) PEFx-300: pancreas of diabetic rats treated with 300 mg/kg body weight. EFx depicting nearly normal islet of langerhans (*green arrows*). (6) PEFx-400: sections of pancreas of diabetic treated rats with 400 mg/kg body weight. EFx showing normal islet of langerhans with numerous beta cells (*green arrows*). (7) PGLIM: pancreatic section of diabetic rats treated with Glibenclamide showing normal pancreatic islet of langerhans with enhancement in the number of beta cells (*dark yellow arrow*).

#### Liver

The liver cells of normal control groups showed eminent hepatocytes with central vein along with portal triad (Figure 10). The damage to the liver cells in the form of damaged central vein, hepatocytes and portal trial could be clearly seen in the group received STZ. The damage to the liver cells were reversed in all the EFx treated groups.

**Figure 10:** Effect of *Euryale ferox salisb* seeds extract (EFx on histological profile of kidney in normal, STZ-induced diabetic untreated and STZ-induced diabetic treated wistar rats (original magnification ×40, DXIT 1200, Nikon, Japan). (1) NKID: heamatoxylin and eosin (H/E) stained sections of kidney of normal control rats showing normal glomeruli with normal baseline and tubules (*yellow arrow*). (2) KSTZ: section of kidney of STZ-induced diabetic rats depicting destroyed glomeruli with fat deposition on baseline along with infiltration of lymphocytes (*red arrows*). (3) KEFx100: kidney section of diabetic rats treated with EFx at dose of 100 mg/kg body weight portraying improved vasculature and glomeruli (*green arrows*). (4) KEFx200: section of kidney of diabetic rats treated with 200 mg/kg body weight of EFx showing normal tubules along with virtually improved structure of glomeruli (*green arrows*). (5) KEFx300: kidney section of diabetic treated rats with 300 mg/kg body weight of EFx depicting nearly normal glomeruli (*green arrows*). (6) KEFx400: section of kidney of diabetic rat received 400 mg/kg body weight of EFx showing normal glomeruli with no infiltration of lymphocytes (*green arrows*). (7) KGLIM: section of kidney of the rat supplemented with Glibenclamide showing normal glomeruli with improved structure of tubules (*dark yellow arrows*).

## Discussion

Acute toxicity study of the methanolic extract demonstrated that different doses of *Euryale ferox salisb*. were non-toxic throughout the experiment. The lethality was found to be zero in the groups received the different doses of *Euryale ferox salisb*. seeds extract. Oral glucose tolerance test studies showed EFx significantly (88.45 ± 0.7672) declined the level of the blood sugar when compared to the glibenclamide (82.80 ± 0.5378). Glibenclamide is often used as insulin stimulant in many studies and also as standard antidiabetic drug in STZ-induced moderate diabetes to compare the antidiabetic potential of various hypoglycemic agents (Andrade et al. 2000). Furthermore, the blood glucose level of STZ-induced diabetic rats was increased to a significant level. EFx treated STZ-induced diabetic rats, lowers the increased blood glucose level to a significant (91.08 ± 0.5402) extent. EFx treated group rats showed improved level of the insulin as compared to the glibenclamide. It has been stated that most of the diabetic complications are mediated through oxidative stress (Matkovics et al. 1997; Kavalali et al. 2003). Studies also suggest involvement of free radicals in pancreatic cell destruction (Lenzen 2008). Histopathological studies of the sections of pancreas, liver and kidney revealed the disturbed morphological features. Islets of langerhans containing β-cells were restored to nearly normal in STZ-induced diabetic treated rats after 45 days of therapy. Distorted central vein and hepatocytes were reinstated to normal in liver of STZ-induced diabetic rats treated with various doses of EFx when compared to the toxic control. Ascending and descending loops were recovered almost to its normal morphological features. All histological changes were well supported with the restored levels of insulin, glucose, glycosylated hemoglobin. Glucose-6-phosphate dehydrogenase (G6PD) is the key enzyme to maintain the blood glucose level (Mayes 2000). In streptozotocin-induced diabetic rats, the reduction of G-6-PDH activity in liver which obstruct glucose utilisation through pentose phosphate pathway as this enzyme activity is controlled by insulin (Ugochukwu and Babady 2003). The plant extract significantly improves this enzyme activity in hepatic tissue which enlighten its another possible way of antidiabetogenic activity. Glucose-6-phosphatase and fructose-1,6-bisphophatase play an important role in glucose homeostasis (Berg et al. 2001). Insulin deficiency results in the activation of gluconeogenic enzymes during diabetes. EFx administration significantly decreased the activity of gluconeogenic enzymes in diabetic rats. The level of plasma insulin was found to increase significantly in diabetic rats treated with EFx, which might be a possible reason for significant reduction in the level of gluconeogenic enzymes. STZ-induced diabetes is characterized by loss in body weight (Al-Shamaony et al. 1994) and this was also observed in the present research exertion. The characteristic loss of body weight is mainly due to increased muscle wasting in diabetes (Swanston-Flatt et al. 1990). *E. ferox salisb*. seeds extract (EFx) and Glibenclamide administration controlled loss of body weight. Hexokinase plays an important role in maintaining the blood glucose homeostasis (Saxena et al. 1992). The activity of hepatic hexokinase was significantly decreased in the STZ-induced diabetic rats. Treatment with different doses of EFx significantly reversed the activity of hexokinase. Increased activity of hexokinase resulted in increased glycolysis which inturn causes improvement in glucose utilization and glycolysis for the production of energy. Oxidative stress has been linked with obesity and insulin resistance, which is recognized by excessive generation of reactive oxygen species (ROS). At present the indicators for evaluation of ROS are the endogenous enzymes such as superoxide dismutase (SOD), catalase (CAT), glutathione Peroxidase (GPx) and glutathione (GSH). Administration of EFx to STZ-induced diabetic rats significantly restored the altered level of antioxidant enzymes in a dose dependent manner. Glycosylation of proteins, oxidative stress and chronic hyperglycemia potentiate the increased risk of cardiovascular diseases through the altered lipid profile. As diabetes is a metabolic disorder, it is characterized not only by increased glucose concentrations but also by altered level of lipid profile. An altered lipid profile was observed with significantly increased concentration of TC, TGs, LDL and HDL and decreased concentration of HDL among diabetic rats (DC) than their normal counterparts. Administration of EFx for 45 days significantly improvised the altered level of TC, TGs. LDL and HDL in a dose dependent manner. Therefore, the plausible mechanism of action of EFx in controlling the blood glucose level might be the enhancement of secretion of insulin from pancreatic β-cells. Furthermore, the mechanism of correction of lipid profile might be due the improved glycogenesis in the liver.

## Conclusion

The above results indicated that *E. Ferox salisb*. seeds extract protect β-cells against ROS-mediated destruction by improvising the levels of antioxidant enzymes and minimizing hyperglycemia which could be due to release of insulin from remnant and recovered β-cells in pancreas in STZ-induced diabetic rats as confirmed by the ultrastructural, histopathological studies. The above research exertion clearly indicates that ethanolic extract of *E. Ferox salisb*. may be utilized as important source of natural antioxidants with antidiabetic and antihyperlipidemic potential and can be used as plausible food additives or as a functional food in future.
